This article has been retracted.

# Ant Colony Optimization-Enabled CNN Deep Learning Technique for Accurate Detection of Cervical Cancer

**DOI:** 10.1155/2023/1742891

**Published:** 2023-02-21

**Authors:** R. Kavitha, D. Kiruba Jothi, K. Saravanan, Mahendra Pratap Swain, José Luis Arias Gonzáles, Rakhi Joshi Bhardwaj, Elijah Adomako

**Affiliations:** ^1^Sri Ram Nallamani Yadava Arts and Science College, Manonmaniam Sundaranar University, Tirunelveli, India; ^2^Department of Information Technology, Sri Ram Nallamani Yadava college of Arts and Science, Manonmaniam Sundaranar University, Tirunelveli, India; ^3^Department of Information Technology, R.M.D. Engineering College, Chennai, India; ^4^Department of Pharmaceutical Sciences and Technology, Birla Institute of Technology, Mesra, Ranchi, India; ^5^Pontificia Universidad Católica del Perú, Peru; ^6^Department of Computer Engineering, Vishwakarma Institute of Technology, Savitribai Phule Pune University, Pune, India; ^7^University of Ghana, Accra, Ghana

## Abstract

Cancer is characterized by abnormal cell growth and proliferation, which are both diagnostic indicators of the disease. When cancerous cells enter one organ, there is a risk that they may spread to adjacent tissues and eventually to other organs. Cancer of the cervix of the uterus often initially manifests itself in the uterine cervix, which is located at the very bottom of the uterus. Both the growth and death of cervical cells are characteristic features of this condition. False-negative results provide a significant moral dilemma since they may cause women to get an incorrect diagnosis of cancer, which in turn can result in the woman's premature death from the disease. False-positive results do not raise any significant ethical concerns; but they do require a patient to go through an expensive and time-consuming treatment process, and they also cause the patient to experience tension and anxiety that is not warranted. In order to detect cervical cancer in its earliest stages in women, a screening procedure known as a Pap test is often performed. This article describes a technique for improving images using Brightness Preserving Dynamic Fuzzy Histogram Equalization. To individual components and find the right area of interest, the fuzzy c-means approach is applied. The images are segmented using the fuzzy c-means method to find the right area of interest. The feature selection algorithm is the ACO algorithm. Following that, categorization is carried out utilizing the CNN, MLP, and ANN algorithms.

## 1. Introduction

Cancer is a disease that is characterized by abnormal cell growth and proliferation. A malignant cell that has invaded an organ has the potential to spread to neighboring tissues and, ultimately, to other organs. Any aberrant cell proliferation, whether benign or malignant, is referred to as a tumor. A benign tumor, like a typical skin wart, remains in its former destination and does not move to other parts of the body or invade neighboring normal tissue. A cancerous tumor, on the other hand, has the ability to both spread throughout the body via the circulatory or lymphatic systems and infiltrate neighboring healthy cells (metastasis). Only malignant tumors are appropriately referred to as cancers, and the danger of cancer stems from its propensity to infiltrate and spread. Cervical cancer first manifests itself in the tissue of the uterine cervix, which is located at the very bottom of the uterus. The infection is characterized by cervical cell growth that is out of control as well as cell death. In about 90 percent of instances of cervical cancer, squamous cell carcinomas are found in the exocervix, which is the region outside of the cervix. Because it is a slow-growing disease that has not yet spread to other regions of the body, cervical cancer in its early stages does not produce any symptoms. Early identification and treatment are both completely curative and preventive when it comes to this condition since it has a prolonged premalignant phase. According to the National Cancer Institute in the United States, cervical cancer is the fourth most frequent illness found in women and is one of the most common causes of cancer death in women worldwide. Cervical cancer is also one of the most common causes of cancer mortality in males [1]. The development of abnormal cells in the cervix's lining is known as cervical cancer. Squamous cell carcinoma is the most typical type of cervical cancer. Cervical cancer symptoms include bleeding after intercourse, in between cycles, or during menopause; watery, red, possibly thick, and foul-smelling vaginal discharge; and pain in the pelvis or during sexual activity. Numerous illnesses were linked to cervical instances. The most common cervical illness among symptomatic southern Ethiopian women was cervical carcinoma. When compared to other cervical cases, the high prevalence of cervical cancer was seen in postmenopausal women. The incidence of cervical cancer [2] and the mortality rate have both decreased in industrialized countries because to the increased use of frequent and mandated screening. On the other hand, cancer is more prevalent in countries with low and moderate incomes, where resources are few and people are not properly educated about the hazards posed by the illness. More women die from cancer in these countries. There are a number of problems associated with automatic screening methods. Particles from the surfaces and surrounding areas of the cervix are carefully extracted during a Pap smear procedure so that they may be inspected under a microscope for cervical cancer or cell changes that could lead to the disease. With a Pap smear, other issues like infections or inflammatory disorders may be found. It is frequently done simultaneously with a pelvic examination and may also be done simultaneously with a test for particular types of human papillomavirus (HPV). These downsides include a decreased sensitivity, uncertainty surrounding cost efficiency, and the inability to detect cases of early abnormalities. It is shown in Figure 1.

The question of whether or not to utilize an automated screening system as opposed to a manual screening method has been hotly contested for decades, and the issue has not been addressed to anyone's satisfaction. They look for early sickness detection, first before indications emerge. This has the advantage of allowing for much early medical intervention for the illness. A problem should only be treated early if doing so leads to a better health outcome than delaying treatment. It has been passionately debated for decades whether to use an automated screening system instead of a manual screening technique, and the problem has not been resolved to everyone's satisfaction. Pathologists are required to examine each subimage on a separate slide under a microscope in the event of manually screening of Pap smear pictures in order to make a medical diagnosis. In the case of manual screening of Pap smear photos, pathologists are required to inspect each subimage on a separate slide under a microscope in order to arrive at a diagnosis of sickness. During mass screening operations, a large number of samples need to be analyzed, which requires more cytotechnicians with higher expertise as well as additional time. The quality of medical photographs has significantly increased because of the developments in medical imaging technology, which has made it possible to diagnose sickness at an earlier stage [3, 4].

Screening may be performed by an automated diagnostic tool without the introduction of observer bias if healthy samples are correctly classified as normal and those with sickness are correctly classified as abnormal. In the event that a patient is given an incorrect diagnosis during screening, they may be subjected to unnecessary follow-up and treatment even when they do not really have the condition. If a test has a false-negative or false-positive result, the one who has the ailment will interpret the result as normal, whereas the individual who does not have the illness would interpret the result as abnormal. Negative smear tests were examined to assess the diagnostic accuracy of recurrence. A total of 122 negative smear results were obtained from women who did not have cervix disease, and 61 of them came form 41 women whose negative smear results were reported within 5.5 years of their CC diagnosis (used as control group). At review, it was discovered that every test from a woman without cervical cancer came back negative. On the other hand, 27.1% of cancer cases from cytologists were recoded as positive. As a direct consequence of this, patients often report feeling of anxiety and depression [5, 6].  Figure 2 shows the different stages of cervical cancer that can be seen in the patients.

Patients who have precancerous lesions will get treatment as quickly as feasible utilizing computer-assisted screening technologies. These approaches have the potential to discover abnormal Pap smear results in patients. The success of an automated screening product is limited by the high cost of the screening equipment, the price of screening activities, and the challenge of achieving high accuracy while simultaneously minimizing the number of false-negative samples produced. It is necessary to develop classification strategies that are both effective and trustworthy if automated systems are to be capable of correctly distinguishing between diseased and healthy samples. Screening samples may now be done more quickly, consistently, and accurately than ever before with the use of machine learning algorithms and medical image processing techniques, all at a cheaper cost than traditional visual screening methods [7]. The precancer stages of cervical cancer are shown in Figure 3.

Image collection, noise reduction, segmentation of regions of interest, feature extraction, and classification are among the major procedures that comprise a Pap smear screening system. The key steps is the Pap smear screening technique. There may be further processes as well. There are several stages to the design process, and each one must be completed successfully for the classification and diagnosis of illness to be done appropriately. False-negative test results are a significant ethical consideration since they can result in a wrong diagnosis of female cancer, which could cause the patient to pass away from the condition. Untrue tests do not provide a severe ethical dilemma, but they do subject the patient to an expensive treatment method and undue anxiety. Other steps may also be included. The process of design consists of multiple steps, and the successful completion of each stage is essential for correctly classifying and diagnosing sickness. False-negative test results are a major ethical concern since they may lead to the incorrect diagnosis of cancer in women, which can then result in the patient's death from the disease. False-positive results do not raise a serious ethical issue; but they do require a patient to undergo an expensive therapeutic process which causes the patient to experience unnecessary worry. It is of the utmost importance to develop a computer-aided diagnosis approach for cervical cancer treatment, in particular in developing countries and poorer nations, where the incidence and fatality rates of the disease are much greater than in wealthy nations.

Researchers are increasingly turning to machine learning (ML), a research approach that is in the process of undergoing fast development. Their goal is to improve cancer detection and treatment. It falls under the umbrella of “artificial intelligence.” Software applications are capable of predicting events more correctly without specific guidelines thanks to machine learning (ML), a type of artificial intelligence (AI). Machine learning algorithms take previous information as input and estimate future accurate output. Medical experts may quickly gain a new viewpoint thanks to the ML categorization of cancer. In reality, the use of machine learning methods may broaden the tumor prognosis window. The ML classification of cancer might provide medical professionals a different perspective in a very short amount of time. The use of machine learning algorithms may, in fact, broaden the scope of cancer prediction [8].

The classification power of ML is most beneficial in biological applications when it is employed in combination with genomic and proteomic data. Because of the growing amount of data available on cancer, machine learning is often used in the process of identifying and diagnosing cancer. The ML approach is reflective of the rising trend toward personalized and predictive medicine in medicine generally.

This article contains a methodology that uses Brightness Preserving Dynamic Fuzzy Histogram. For improving image contrast, fuzzy logic-based histogram equalization (FHE) is suggested. As opposed to conventional crisp histograms, fuzzy histograms are built using fuzzy set theory in order to more effectively handle the ambiguity of grey level data. The fuzzy distribution is divided into two subhistograms based on the median value of the original image in the second stage, and each subhistogram is then separately balanced to preserve contrast enhancement. Two well-known metrics utilized to assess the both qualitative and quantitative assessments of the proposed FHE approach are average information contents (AIC) and natural image quality evaluator (NIQE) index for different pictures. Equalization for image enhancement. Images are segmented to detect correct region of interest using the fuzzy c-means technique. In this method, the author transformed the colour image to grayscale and applied a median filter to lessen the level of noise and improve the representation of the image before using the fuzzy c-means clustering algorithm. Clusters and classification are the third and fourth steps of this process, respectfully. The centre value may be calculated thanks to the patch-based sorting. A data collection is divided into *N* clusters using the fuzzy c-means (FCM) data clustering method, with each data point in the dataset to some extent belonging to each cluster. A data point will have a high degree of membership in a cluster, for instance, if it is near to the cluster's center. ACO algorithm is used for feature selection. Then, classification is performed using CNN, MLP, and ANN algorithms. Accuracy of ACO-CNN is highest among all classifiers used in this experimental study.

Both aberrant cell growth and reproduction, which are both diagnostic indications of the illness, are characteristics of cancer. The membrane of the uterine cervix, which is found at the base of the uterus, is where cervical cancer first shows symptoms. Cell death and uncontrollable cervical cell proliferation are symptoms of the illness. The fourth most prevalent disease in women and one of the leading causes of cancer-related deaths in women globally is cervical cancer.

The remainder of this paper is organized as follows: Section 2 covers the literature survey.  Section 3 covers the methodologies, and the results are analyzed in Section 4.  Section 5 contains concluding remarks as well as future scope of the research.

## 2. Literature Survey

The augmentation of a photograph is done with the intention of calling attention to certain aspects in order to facilitate future research. A machine learning-based programme called automated visual assessment (AVE) scans digital images of the cervix for indications of cancer or precancer. An AVE-positive result indicates the existence of troubling lesions that are either suggestive of cancer or enhance the possibility that cancer will develop in the near future. An AVE-negative outcome, on the other hand, indicates a cervix that is not at higher risk for cancer. The methodologies may be broken down into two primary categories: the spatial domain and the frequency domain. The values of a picture's pixels are inputted directly into mathematical calculations that are performed in the spatial domain. The picture is transformed using a Fourier transformation in the frequency domain first, and then, the inverse of the image that was converted using the Fourier transform is used to create the final image. Filtering is one component of image enhancement, and its purposes include reducing distracting noise and bringing attention to certain aspects of an image.

The authors Lu et al. [8] offered a comparative analysis of a variety of techniques for improving the quality of the pictures. Approaches from the spatial domain, the frequency domain, and the fuzzy domain were all used throughout the investigation. Approaches based on histograms and fuzzy logic have both been shown to be effective. The author of the research believes that the evaluation of the fuzzy-based enhancement's *K* factor might perhaps be automated by employing ant colony optimization to provide a more accurate representation of the image.

According to the author, the Poisson noise is introduced into cell images as a result of the noneven distribution of photons. According to the findings of the study, an adaptive Wiener filter has the potential to effectively minimize the Poisson noise. Even if the picture qualities change from one location to another, it is still feasible to denoise photographs by using an adaptive Wiener filter [9].

Bihistogram equalization is a method that was created by Tang and Isa [10] with the purpose of increasing the quality of grayscale pictures. The input histogram is used to generate not one but two subhistograms. The picture's oversaturation was brought under control by clipping the histogram, and then, the output that was generated was equalized and mixed to make the finished product. In general, the performance of the authors' technique is superior to that of existing histogram-based improvement algorithms, as shown by a comparison with those algorithms.

It was found by Kumbhar et al. [11] that the main attributes of an image may be retrieved for enhanced diagnosis if the features of medial photos are increased. The images were run through filters before any sharpening or noise reduction methods were applied to them. In addition to that, an effect called “Adaptive Histogram Equalization and Average Filter” was added to the photo in order to make it seem better.

In the Herlev dataset, Chankong et al. [12] segregated the nucleus from the cytoplasm by using a patch-based version of the fuzzy c-means clustering algorithm. In this method, the author converted the colour image to grayscale and used a median filter to reduce the amount of noise and smooth out the appearance of the picture. The third and fourth processes in this process are called clustering and segmentation, respectively. The patch-based sorting allowed for the calculation of the central value.

According to Sharma and Mangat [13], an additional improvement was made to the work, and the author improved the “fuzzy c-means (FCM)” clustering technique by working with various numbers of clusters rather of just one. This was done in order to reinforce the clustering of the data. The author recommended combining techniques to segmentation with methods for locating areas of interest in order to improve the accuracy of the segmentation process. There is a possibility that the present accuracy of the Herlev dataset may be improved using a variety of feature variations, improved noise reduction techniques, and segmentation methods (93.7 percent).

Saha et al. [14] introduced a circularly shaped function that put a restriction on the form of the cluster in order to enhance the border of the nucleus. This was done in order to make the nucleus seem more complete.

A categorization system that is based on texture and was created by Mariarputham and Stephen [15] is used to categorize smear photographs into a total of seven separate groups. In terms of the accuracy of classification, it was shown that SVM had a precision of 97.38 percent for normal squamous, 93.89 percent for intermediate squamous, 87.33 percent for mild dysplasia, and 58.52 percent for severe dysplasia. The RBF, linear, and quadratic SVM kernels were used in the classification process.

A wide range of neural network architectures were put to the test by Devi et al. [16] for the purpose of disease diagnosis. ANN designs such as the multilayered perceptron may be helpful when it comes to the acceleration of the detection process. Both a feedforward network and a knowledge-based neural network were utilized in order to map the input pictures with the rules and extract the features that are necessary for classification. As a result, the classification results exhibited by the network were superior, and it had a decent accuracy rate. The results of the classification carried out using the artificial neural network (ANN) method are better and have a high rate of accuracy.

Athinarayanan et al. [17] developed a categorization system for cervical disease by analyzing images obtained from Pap smears. In order to improve the rough set text on cooccurrence matrix, we made use of the ERSTCM and CABS descriptors as well as the concatenated feature extraction approach (CFE). Using a classifier, it is possible to measure the performance of the extracted features by comparing them to statistical criteria such as sensitivity, specificity, and accuracy. This can be done with the help of a classification algorithm (FL-HKSVM). The performance of the concatenated feature extraction method was superior than that of the other two classifiers. Feature extraction is the process of converting raw data into manageable quantitative properties while conserving the original dataset's characteristics. It yields superior results when compared to utilizing machine learning on the raw data directly. Since CNNs can automatically generate features from time series information and frequency represented images, they are most frequently employed in healthcare applications. After that, a classifier network uses these features to do classification and regression. A neural network that has hundreds of hidden layers is referred to as a deep learning network. This kind of network is able to capture the nonlinear link that exists between intricate patterns and make accurate predictions. For the purposes of picture recognition and analysis, deep neural network topologies such as the convolution neural network (CNN) are often used [18]. A system will automatically learn features at many different levels of abstraction in order for it to be able to learn every conceivable characteristic. This is necessary for the system to be able to learn everything.

The precision of the cell segmentation is a crucial component in the overall success of the traditional machine learning approaches. Taha et al. [19] proposed a technique for categorizing cells without the need for segmentation. Their approach included the use of a deep feature learning convolution neural network. They were successful in assigning categories to the Herlev dataset with a rate of accuracy of 98 percent, which is an admirable achievement.

Hyeon et al. [20] trained a model that can differentiate between healthy and sick cervical cells by using a convolutional neural network (CNN) and retrieving feature vectors from images of cervical cells. These collected characteristics were trained with the use of an SVM classifier, which resulted in a success rate of 78 percent overall. The study presented here proposes a classification model for prostate cancer that makes use of deep learning methods and achieves an accuracy of 80.1% on training sets and 78.1% on testing sets, respectively.

Devi et al. [16] investigated a variety of neural network architectures, convolutional neural network architecture, and feedforward network architecture. According to the results, the performance of ANN might be enhanced by including a learning capacity that assists in the improvement of its efficiency through the evaluation of exceptional performance.

## 3. Methodology

This article contains a methodology that uses Brightness Preserving Dynamic Fuzzy Histogram Equalization for image enhancement. Images are segmented to detect correct region of interest using the fuzzy c-means technique. ACO algorithm is used for feature selection. Then, classification is performed using CNN, MLP, and ANN algorithms. Accuracy of ACO-CNN is highest among all classifiers used in this experimental study. Interstrategies modelled after ants are referred to as “ants.” Biological ants' pheromone-based communication is frequently the dominating paradigm. For many optimization projects requiring some kind of graph, local search algorithms combined with artificial ants have emerged as the preferred approach. This framework is shown in Figure 4.

By using the technique for fuzzy histogram equalization, the method known as “Brightness Preserving Dynamic Fuzzy Histogram Equalization” has been updated in order to increase both its brightness and its contrast. It was chosen to first use a Gaussian kernel to smooth out the image histogram and then to segment the troughs for dynamic equalization. This was done after the decision was made. Histograms are processed using crisp histograms so that the contrast may be made better. Brightness Preserving Dynamic Fuzzy Histogram Equalization [21] is a modified method that was developed as a result of the authors' use of fuzzy statistics in the original methodology. As a result, the authors were able to efficiently keep the mean image brightness.

The fuzzy c-means clustering approach combines pixels and groups together according to the similarity criteria that they share with one another. Because the nucleus and cytoplasm both have consistent pixel values, this method was successful when applied to Pap smear photographs. When an algorithm uses fuzzy c, it indicates that it does not definitively decide on the absolute membership value of a certain cluster. Because it takes into consideration the degree of membership and then utilizes that value to identify the cluster, it is possible to accomplish an accurate segmentation using this method. In order to do medical image analysis, one of the most important steps is to cut the image into a number of smaller, more manageable pieces. Because of its accuracy and ease of use, the fuzzy c-means method is a popular choice for clustering data in the field of medical image analysis [22].

The selection strategy is used to both increase the dimensionality of the input and recover the prominent aspects of the sign representation. Within this part, ant colony optimization, often known as ACO, is used as a tool to assist in the process of feature selection. Finding good pathways throughout graphs is a computer challenge that can be solved using the probability ant colony optimization algorithm (ACO). Multiagent techniques influenced by the behavior of actual ants are represented by artificial ants. Biological ants' pheromone-based communication is frequently the dominating paradigm. Combinations of artificial ants and local search algorithms have become the standard method for several optimization tasks that involve networks, such as route choice and internet routing. According to ACO, which is one of the most recent approaches to approximation optimization, actual ants, which use the chemical signaling agent known as pheromone to communicate with one another, may use to find the shortest pathways between their nest and food sources. Pheromones are used by ants to communicate with one another [23].

The efficacy of machine learning methods is severely limited when they are used to enormous datasets because of challenges such as underfitting, model complexity, and a lack of resource optimization. These challenges make it difficult for the approaches to be effective. Deep learning networks may be applied to massive amounts of data in order to discover new information, make predictions about the future based on that knowledge, and put that knowledge to use. The machine models are able to learn directly from photographs, videos, and text thanks to a technique called deep learning. As the amount of data available increases, several deep learning architectures have been implemented in order to obtain an outstanding level of performance in comparison to previous machine learning methods. The approach known as “Brightness Preserving Dynamic Fuzzy Histogram Equalization” has been revised to increase both brightness and contrast utilizing the fuzzy histogram equalization technique. The fuzzy c-means clustering method groups and mixes pixels in accordance with the similarity criteria they share. This technique worked well with Pap smear images since the nucleus and cytoplasm both have constant pixel values.

The convolutional neural network is a deep neural network that is extensively used in computer vision. It is constructed by assembling deep neural network design. CNN is built on many different layers, including convolutional, pooling, activation, and linked convolutional layers. A deep convolutional neural network (CNN) is an end-to-end architecture that, as the name indicates, is composed of a number of convolutional layers. The filters that are used in the convolutional layer are the most essential component there. At the convolutional layer, just a small number of the input picture's pixels—let us say 3 × 3—are allowed to get through the filter [24].

The values of the pixels are subjected to a “dot” operation, and the filter uses a predetermined weight to determine how much of an impact this operation will have on the final result. As a direct consequence of this procedure, the convolutional layer will provide an image with a more compact matrix containing the data points. The activation layer takes the shape of a matrix and is responsible for supplying the network with nonlinearity as well as back propagation. Pooling decreases the number of layers in samples, in addition to lowering the size of the filter matrix. The selection of a single feature from each group by the pooling layer gives rise to the name “max layer,” which describes this selection. The max layers are linked to provide a list of probabilities for a variety of probable labels for the image that is being analyzed. When making a decision on how to classify anything, the label that seems to fit best is the one that is chosen.

It was Professors Bernard Widrow and Ted Hoff, back in 1960, who created a mathematical model. Information may be processed in an analogous manner to the way the human brain works. Using this strategy, researchers were able to classify and forecast chronic illnesses like breast cancer. ANN [25] is a powerful tool for revealing BC's simple connections. An ML process was used to create and construct this algorithm for a specific purpose, such as pattern cataloguing. Edges of the ANN model refer to the connections made between layers. Input, intermediate, and output layers are formed by the arrangement of neurons. Edges link the neurons, and each side has a vertex, which is termed “wait” in this context. The underlying concept of ANN is that of a network of neurons.

An MLP algorithm is a kind of machine learning algorithm that recreates the decision-making and learning processes of a natural artificial neural network (ANN) by using several fully connected layers. MLP used three different layers for its nodes: (A) the initial layer, also known as the input layer; (B) the intermediate layer, also known as the hidden layer; and (C) the output layer. The back propagation method is used in order to affect an update to the weight of the MLP. MLP allows for the recognition of nonlinear datasets that are separable [26].

## 4. Result Analysis

The Herlev dataset consists of 242 normal cells, 650 images are used to train the model, and the remaining 267 images were used to test the model [27]. A model's performance can be gauged by its sensitivity and specificity. In contrast to specificity, which measures how well the model predicts real negatives, sensitivity measures how well the model predicts true positives. The results are shown in Figure 5.

Brightness Preserving Dynamic Fuzzy Histogram Equalization is used for image enhancement. Images are segmented to detect correct region of interest using the fuzzy c-means technique. ACO algorithm is used for feature selection. Then, classification is performed using CNN, MLP, and ANN algorithms. Accuracy of ACO-CNN is highest among all classifiers used in this experimental study. Various authors have investigated similar studies in their results. The result trend of the current study is similar to the findings of various researchers. A deep learning method for cervical cancer detection using Pap smear images is proposed by Taha et al. [19]. They use the Herlev public database for single cell Pap smears to demonstrate the effectiveness of this novel approach, and the results of the experiments show that our suggested system works noticeably better than other cutting edge techniques.

## 5. Conclusion

Since abnormal cell growth and multiplication are diagnostic signs of cancer, this condition is regarded as its distinguishing feature. Once malignant cells have invaded an organ, it is possible that they will spread to the tissues nearby before eventually reaching other organs. The uterus cervix, which is located at the very bottom of the uterus, is frequently where uterine cervical cancer first manifests itself. Both the growth and death of cervical cells are hallmarks of this condition. Both of these procedures are signs. False-negative results pose a huge ethical problem since they may result in women being given the wrong cancer diagnosis, which may cause the woman to pass away from the disease too soon. In this sense, erroneous negative outcomes might be to blame for the early demise of females. False-positive results do not lead to any significant ethical issues, but they do make a patient undergo an expensive and time-consuming treatment process, as well as put them through unneeded stress and concern. Women are frequently subjected to a monitoring procedure called a Pap test in an effort to find cervical cancer in its earliest stages, when it is most curable. By using the procedures described in this article, which make use of a method called Brightness Preserving Dynamic Fuzzy Histogram Equalization, image quality can be enhanced. Images are segmented using the fuzzy c-means technique to determine the proper area of interest. The ACO algorithm is used to select the characteristics. Then, classification is performed with the aid of the CNN, MLP, and ANN algorithms. Of all the classifiers used in this experimental inquiry, the ACO-CNN classifier had the highest accuracy.

## Figures and Tables

**Figure 1:** Cervical cancer symptoms.

**Figure 2:** Stages of cervical cancer.

**Figure 3:** Cervical precancer stages.

**Figure 4:** Ant colony optimization-enabled CNN deep learning technique for accurate detection of cervical cancer.

**Figure 5:** Accuracy, sensitivity, and specificity of machine learning techniques for diagnosis of cervical cancer on the Herlev dataset.

## Data Availability

The corresponding author will provide data on request.

## References

[1] Shafabakhsh R., Reiter R. J., Mirzaei H., Teymoordash S. N., Asemi Z. (2019). Melatonin: a new inhibitor agent for cervical cancer treatment. *Journal of Cellular Physiology*.

[2] US Preventive Services Task Force, Curry S. J., Krist A. H. (2018). Screening for cervical cancer. *Journal of the American Medical Association*.

[3] Pankaj S., Nazneen S., Kumari S. (2018). Comparison of conventional Pap smear and liquid-based cytology: a study of cervical cancer screening at a tertiary care center in Bihar. *Indian Journal of Cancer*.

[4] Zamani A. S., Anand L., Rane K. P. (2022). Performance of machine learning and image processing in plant leaf disease detection. *Journal of Food Quality*.

[5] Dong N., Zhao L., Wu C. H., Chang J. F. (2020). Inception v3 based cervical cell classification combined with artificially extracted features. *Applied Soft Computing*.

[6] Veluri R., Patra I., Naved M. (2022). Learning analytics using deep learning techniques for efficiently managing educational institutes. *Materials Today: Proceedings*.

[7] Zhang T., Luo Y. M., Li P. (2020). Cervical precancerous lesions classification using pre-trained densely connected convolutional networks with colposcopy images. *Biomedical Signal Processing and Control*.

[8] Lu J., Song E., Ghoneim A., Alrashoud M. (2020). Machine learning for assisting cervical cancer diagnosis: an ensemble approach. *Future Generation Computer Systems*.

[9] Deepa T., Rao A. N. (2016). A study on denoising of poisson noise in Pap smear microscopic image. *Indian Journal of Science and Technology*.

[10] Tang J. R., Isa N. A. M. (2014). Adaptive image enhancement based on bi-histogram equalization with a clipping limit. *Computers & Electrical Engineering*.

[11] Kumbhar U., Patil V., Rudrakshi S. (2013). Enhancement of medical images using image processing in matlab. *International Journal of Engineering Research and Technology*.

[12] Chankong T., Theera-Umpon N., Auephanwiriyakul S. (2014). Automatic cervical cell segmentation and classification in Pap smears. *Computer Methods and Programs in Biomedicine*.

[13] Sharma B., Mangat K. K. (2016). Various techniques for classification and segmentation of cervical cell images-a review. *International Journal of Computer Applications*.

[14] Saha R., Bajger M., Lee G. Spatial shape constrained fuzzy c-means (fcm) clustering for nucleus segmentation in Pap smear images.

[15] Mariarputham E. J., Stephen A. (2015). Nominated texture based cervical cancer classification. *Computational and Mathematical Methods in Medicine*.

[16] Devi M. A., Ravi S., Vaishnavi J., Punitha S. (2016). Classification of cervical cancer using artificial neural networks. *Procedia Computer Science*.

[17] Athinarayanan S., Srinath M., Kavitha R. (2016). Computer aided diagnosis for detection and stage identification of cervical cancer by using Pap smear screening test images. *ICTACT Journal on Image & Video Processing*.

[18] Zhang L., Lu L., Nogues I., Summers R. M., Liu S., Yao J. (2017). DeepPap: deep convolutional networks for cervical cell classification. *IEEE Journal of Biomedical and Health Informatics*.

[19] Taha B., Dias J., Werghi N. Classification of cervical-cancer using Pap-smear images: a convolutional neural network approach.

[20] Hyeon J., Choi H.-J., Lee K. N., Lee B. D. Automating papanicolaou test using deep convolutional activation feature.

[21] Sheet D., Garud H., Suveer A., Mahadevappa M., Chatterjee J. (2010). Brightness preserving dynamic fuzzy histogram equalization. *IEEE Transactions on Consumer Electronics*.

[22] Tang J. R., Mat Isa N. A., Ch’ng E. S. (2015). A fuzzy-c-means-clustering approach: quantifying chromatin pattern of non-neoplastic cervical squamous cells. *PLoS One*.

[23] Singh S., Janghel R. R., Karuppusamy P., Perikos I., García Márquez F. P. (2022). Early diagnosis of Alzheimer’s disease using ACO optimized deep CNN classifier. *Ubiquitous Intelligent Systems. Smart Innovation, Systems and Technologies*.

[24] Ghoneim A., Muhammad G., Hossain M. S. (2020). Cervical cancer classification using convolutional neural networks and extreme learning machines. *Future Generation Computer Systems*.

[25] Zhang J., Li C., Yin Y., Zhang J., Grzegorzek M. (2023). Applications of artificial neural networks in microorganism image analysis: a comprehensive review from conventional multilayer perceptron to popular convolutional neural network and potential visual transformer. *Artificial Intelligence Review*.

[26] Balaha H. M., Shaban A. O., el-Gendy E. M., Saafan M. M. (2022). A multi-variate heart disease optimization and recognition framework. *Neural Computing and Applications*.

[27] Jantzen J., Dounias G. (2006). Analysis of Pap-smear image data. *Nature-Inspired Smart Information Systems 2nd Annual Symposium*.

